# Computer-Aided Multiclass Classification of Corn from Corn Images Integrating Deep Feature Extraction

**DOI:** 10.1155/2022/2062944

**Published:** 2022-08-10

**Authors:** Bhamidipati Kishore, Ali Yasar, Yavuz Selim Taspinar, Ramazan Kursun, Ilkay Cinar, Venkatesh Gauri Shankar, Murat Koklu, Isaac Ofori

**Affiliations:** ^1^Department of Computer Science and Engineering, Manipal Institute of Technology, Manipal Academy of Higher Education, Manipal, Karnataka 576104, India; ^2^Department of Mechatronic Engineering, Selcuk University, Konya, Turkey; ^3^Doganhisar Vocational School, Selcuk University, Konya, Turkey; ^4^Guneysinir Vocational School, Selcuk University, Konya, Turkey; ^5^Department of Computer Engineering, Selcuk University, Konya, Turkey; ^6^Manipal University Jaipur, Jaipur, Rajasthan, India; ^7^Department of Environmental and Safety Engineering, University of Mines and Technology, Tarkwa, Ghana

## Abstract

Corn has great importance in terms of production in the field of agriculture and animal feed. Obtaining pure corn seeds in corn production is quite significant for seed quality. For this reason, the distinction of corn seeds that have numerous varieties plays an essential role in marketing. This study was conducted with 14,469 images of BT6470, Calipso, Es_Armandi, and Hiva types of corn licensed by BIOTEK. The classification of images was carried out in three stages. At the first stage, deep feature extraction of the four types of corn images was performed with the pretrained CNN model SqueezeNet 1000 deep features were obtained for each image. In the second stage, in order to reduce these features obtained from deep feature extraction with SqueezeNet, separate feature selection processes were performed with the Bat Optimization (BA), Whale Optimization (WOA), and Gray Wolf Optimization (GWO) algorithms among optimization algorithms. Finally, in the last stage, the features obtained from the first and second stages were classified by using the machine learning methods Decision Tree (DT), Naive Bayes (NB), multi-class Support Vector Machine (mSVM), k-Nearest Neighbor (KNN), and Neural Network (NN). In the classification processes of the features obtained in the first stage, the mSVM model has achieved the highest classification success with 89.40%. In the second stage, as a result of the classifications performed through the active features selected by using three types of feature selection algorithms (BA, WOA, GWO), the classification success obtained with the mSVM model was 88.82%, 88.72%, and 88.95%, respectively. The classification accuracies of the tested methods and the classification accuracies obtained in the first stage are close to each other in terms of classification success. However, with the algorithms used in feature selection, successful classification processes have been carried out with fewer features and in a shorter time. The results of the study, in which classification was carried out in the inexpensive, the objective, and the shorter time of processing for the corn types, present a different perspective in terms of classification performance.

## 1. Introduction

Corn, one of the basic grain products, is a staple food for millions of people all over the world, particularly in Latin America, Asia, and Africa. Corn is used by being processed in various food products directly as human food such as corn flour, semolina, starch, snacks, breakfast cereals as well as it is used in the production of animal feed [1]. Corn, or maize, which can be harvested once a year, is an agricultural product that ranks third after wheat and rice in terms of cultivation area throughout the world [2]. As a multipurpose grain widely cultivated in many parts of the world, corn has many different types across the world [3]. The distinction of corn type is of great importance for crop monitoring, high-throughput phenotyping, and yield prediction [4]. The region where it is grown has a strong influence on the quality and commercial value of corn. Hence, as the geography changes, the unique characteristics of corn also differ [5]. To the extent that the classification of corn has an impact on the final product and its quality, it plays an important and critical role in determining the market value. The main purpose of classification is to facilitate the correct commercialization of corn, as well as to provide information about the storage and processing [6]. Seed purity is an important parameter for the evaluation of seed quality and can be effectively examined by the seed classification [7]. In addition to the fact that there are numerous literature studies conducted in this field, it is also seen that classification studies are carried out in agricultural products.

In recent years, multispectral and hyperspectral imaging techniques have been used as well as several image processing, deep learning, and machine learning methods for the classification and quality evaluation of corn. When the literature in this area is examined, it is seen that the classification of corn has been performed with Multi-Linear Discriminant Analysis (MLDA) and Least-Squares Support-Vector Machine (LS-SVM) [7], Radial Basis Function Neural Network (RBFNN) and SVM [8], Principal Component Analysis + Partial Least Squares Discriminant Analysis (PCA + PLS-DA) [6], and Deep Convolutional Neural Network (DCNN) [9].  Table 1 gives the results of grain products' classification with various artificial intelligence methods and the results of these classifications.

The aim of this study is to compare nondestructive classification models by using the images of different corn types. A limited number of features can be obtained by extracting color, morphological, and shape features from corn grain images. However, a large number of features are obtained with Deep Feature Extraction. The deep learning model tested and used in the study is based on the SqueezeNet architecture as it has a smaller structure compared to well-known pretrained network designs [10]. The created model was used to extract the deep features of the images. Different classification models have been created to classify these extracted features. Decision Tree (DT), Naive Bayes (NB), Multi-Class Support Vector Machine (mSVM), k-Nearest Neighbor (KNN), and Neural Network (NN) classifiers [11–16] were used in these models. Among the deep features, the more effective features were selected with the meta-heuristic algorithms, Bat Algorithm (BA), Whale Optimization Algorithm (WOA), and Gray Wolf Optimization (GWO) [16–20]. Furthermore, the selected features were classified by machine learning algorithms DT, NB, mSVM, KNN, and NN. 10-fold cross validation was used to objectively measure the success of the models.

The main contributions of this research to the literature are listed below:

1. A different approach based on deep feature extraction, selection, and classification strategy is presented for the classification of corn types used in the study.
2. The deep features of the corn images were extracted and classified with DT, NB, mSVM, KNN, and NN models.
3. The features obtained as a result of the most effective features' selection process with BA, WOA, and GWO were classified with DT, NB, mSVM, KNN, and NN models.
4. As a result of the processes, the classification success of all models, as well as the classification times, were compared and the optimum classification model was determined.

In order to realize the abovementioned contributions, the article is organized as follows: in Section 2, the materials and methods used in this research are described. In Section 3, the experimental results for the multiple classification problem are presented. In Section 4, the performance of the proposed framework is evaluated.

## 2. Material and Methods

### 2.1. Dataset

In this study, the licensed BT6470, Calipos, Es_Armandi, and Hiva types belonging to BIOTEK were used. A total of 14,469 corn seeds images were obtained from 1-kilogram corn of each type, 3056, 5090, 3385, and 2938, respectively. Each image is 350 × 350 pixels in size. In Figure 1, sample seed images of the corn types in the dataset are given.

### 2.2. Convolutional Neural Network (CNN)

CNN is a deep learning method that has been frequently used in the literature recently, designed to recognize visual patterns directly from image pixels by minimizing preprocessing [21]. CNNs are a kind of feedforward neural network with many layers. In Figure 2, a typical CNN architecture is shown [22].

#### 2.2.1. SqueezeNet

First proposed by Iandola et al. in 2016, SqueezeNet is a specially designed CNN model [23]. It consists of 15 layers as two convolution layers, three maximum pooling layers, eight fire layers, a global average pooling layer, and an output layer softmax. SqueezeNet has a lightweight structure with fewer structural parameters and less computation. SqueezeNet has only 1 × 1 and 3 × 3 convolution cores, and its purpose is to simplify the complexity of the network to achieve the best classification accuracy [24]. At the end of the layers, there are fully connected (FC) layers with average pooling and 1000 neurons.

### 2.3. Feature Selection

Feature selection plays an important role in terms of dimensionality reduction and classification in high-dimensional datasets. In the feature selection process, only the most active features in the datasets are selected. A good feature selection technique aims to improve classification performance while reducing computational cost and time [25]. Searching for the best feature set is a challenging problem in the feature selection process. Metaheuristic algorithms perform well in finding the optimal solution for this type of problem [26]. In this study, BA, WOA, and GWO metaheuristic optimization algorithms were utilized for feature selection.

#### 2.3.1. Bat Optimization Algorithm (BA)

Bat optimization algorithm, which is a metaheuristic optimization method based on the behavior of bats, was proposed by Yang in 2010. It is an optimization algorithm inspired by the behavior of bats to determine the direction and distance of an object by utilizing echolocation [27]. The basics of the bat optimization algorithm are given as follows [28]:

  Rule 1: All bats locate their prey by echolocation.
  Rule 2: Each bat flies randomly in position *x*_*i*_, *v*_*i*_ speed, and *f*_min_ frequency and searches for their prey by varying the wavelength (*λ*) and sound output (A).
  Rule 3: Bats can adjust their wavelength and sound output for different situations.

It is frequently used in feature reduction problems in the feature extraction [29]. Each bat is associated with a set of binary coordinates indicating whether a feature belongs to the final feature set. The feature reduction function, which depends on the number of bats, requires that a classifier with features defined by the position of each bat is trained and evaluated on the classifier set [30].

#### 2.3.2. The Whale Optimization Algorithm (WOA)

Whale Optimization Algorithm (WOA), first brought to the literature by Mirjalili and Lewis in 2016, is a metaheuristic optimization method that mimics the hunting behavior of humpback whales. It finds an area of study in classical engineering problems such as unimodal, multimodal, fixed-dimensional modal, and composite functions. Based on the hunting behavior of whales, this technique has both exploitation and exploration stages with the spiral bubble net attack method. In this respect, it is used for the global optimization target [31, 32]. This technique can be used to find the best subset of features that maximizes classification success while keeping the minimum number of features [33].

#### 2.3.3. Gray Wolf Optimization (GWO)

It is a new metaheuristic optimization method developed by Mirjalili et al. in 2014. The number of group individuals of wolves living as a group varies between 5 and 12. In the gray wolf group, which has a social hierarchy, the alpha wolf, the leader, is followed by the beta and delta wolves. Omega wolves are the lowest-level wolves. In this strategy, gray wolves first recognize the location of the prey and surround it under the leadership of the alpha wolf. In the mathematical model of gray wolves' hunting strategy, it is assumed that alpha, beta, and delta wolves provide better information about prey location. Therefore, the first three best solutions (alpha, beta, delta) are used to update the positions of wolves in the GWO algorithm. For this reason, omega wolves have no place in the algorithm [34, 35]. The features of GWO such as fast convergence, and simple and easy implementation are the reasons for its preference compared to other optimization methods. High-classification success can be achieved with the successful application of feature selection in datasets and a small number of features [36].

### 2.4. Classification Methods

Within the scope of this study, five multiclass supervised classification algorithms are focused, which are DT, NB, mSVM, KNN, and NN methods. The detailed information about each method is given below. The features obtained from deep feature extraction of corn images are given as separate inputs to these methods:

  Decision Tree (DT): The use of Decision Tree algorithms was started first in 1995. The DT method is used to solve regression or classification problems [37].
  Naive Bayes (NB): It is a simple probabilistic algorithm using Bayes' theorem. Naive Bayes performs the classification process by assuming that all variables are independent. This conditional assumption of independence is rarely valid in real-world applications. That is why it is characterized as naive. In spite of this, the algorithm tends to learn quickly in a variety of supervised classification problems [38].
  Multi-Support Vector Machines (mSVM): Support vector machine (SVM) is one of the most powerful kernel-based machine learning tools used for classification and regression problems and it can distinguish all classes with a single optimization process [39, 40].
  K-Nearest Neighbor (KNN): It is one of the frequently used algorithms in the machine learning field due to its versatility and ease of use. However, since KNN uses all the training data, it needs more time in analyzing large data and high memory for storage. The letter “K” indicates the number of nearest neighbors, and the term “nearest neighbor” indicates that the algorithm searches for the nearest point it needs to classify and label the closest point assigned to it [41].
  Neural Network (NN): It is a mathematical system consisting of many processing units (neurons) interconnected in a weighted manner. Unlike other statistical, mathematical, and experimental techniques that require prior knowledge, the NN model performs classification processes by using the similarities and relationships between the data [42].

### 2.5. K-Fold Cross Validation

The standard *k* folds operation divides the data into *k* subsets. Each fold contains approximately an equal number of data, and fold membership is randomly assigned typically. If the dataset is relatively small, stratified random sampling is also used to ensure that the target variable is approximately uniformly distributed in each fold. After dividing the data into *k* folds, the candidate model is then subjected to an iterative evaluation process. During iteration, each fold is used to train the *k* − 1 candidate model and the performance of the model is measured with the remaining fold. This process is repeated until each fold is fully used as a validation set, and a total of *k* retraining and validation processes are performed for each candidate model [43–46].  Figure 3 shows the *k* = 10 fold cross-validation process used in the study.

### 2.6. Evaluation Metrics

In order to objectively evaluate the performance of the methods, Accuracy (ACC), Sensitivity (TPR), Specificity (TNR), Precision (PRE), F1-Score, and Mathew Correlation Coefficient (MCC) metrics are calculated from the confusion matrix[11, 47–50]. In Figure 4, a multiclass confusion matrix is shown. The performance metric calculations are given in equations (1)–(6).

(1) $$\begin{array}{c} \text{Accuracy}\left(\text{ACC}\right)=\frac{\text{TP}+\text{TN}}{\text{TP}+\text{TN}+\text{FP}+\text{FN}}, \end{array}$$

(2) $$\begin{array}{c} \text{Sensivity}\left(TPR\right)=\frac{\text{TP}}{\text{TP}+\text{FN}}, \end{array}$$

(3) $$\begin{array}{c} \text{Specificity}\left(TNR\right)=\;\frac{\text{TN}}{\text{TN}+\text{FP}}, \end{array}$$

(4) $$\begin{array}{c} \text{Precision}=\left(PRE\right)\frac{\text{TP}}{\text{TP}+\text{FP}}, \end{array}$$

(5) $$\begin{array}{c} F1-\text{Score}=2*\frac{\text{Sensivity}*\text{Precision}}{\text{Sensivity}+\text{Precision}}, \end{array}$$

(6) $$\begin{array}{c} \text{Mathew Correlation coefficient}\left(MCC\right)=\frac{\text{TP}*\text{TN}-\text{FP}*\text{FN}}{\sqrt{\left(TP+FN\right)+\left(TP+FP\right)+\left(FN+TN\right)\left(FP+TN\right)}}. \end{array}$$

## 3. Experimental Results and Discussion

A computer with Intel (*R*) Core (TM) i7-10750H CPU @ 2.60 GHz and 32 GB RAM (3200 MHz) was used for this study. First, as a result of deep feature extraction of 14,469 corn images with the pre-trained SqueezeNet CNN model, a feature vector of 14,469 × 1000 was obtained with 1000 features obtained from each image. In the classification of these feature vectors, machine-learning methods (DT, NB, mSVM, KNN, NN) were used as classifiers. The 10-fold cross-validation method was used to evaluate the success of the classification models. Among the deep features extracted from SqueezeNet, more effective features were selected via BA, WOA, and GWO optimization techniques. The parameters of optimization algorithms (BA, WOA, GWO) used in feature selection and (mSVM) techniques used as classifiers are given in Table 2.

The feature vectors obtained from the feature selection were reclassified with the specified classification methods as in the first step, and the 10-fold cross-validation method was used again to evaluate the success of the models. The general block diagram of the study is given in Figure 5.

The classification performances of the feature vector obtained from deep feature extraction of corn images and feature vector obtained after feature selection were calculated separately.  Table 3 gives the classification performances and the number of features obtained.

According to Table 3, the mSVM is the most successful model as a result of the classification performed with 1000 features. The mSVM model is followed by NN, KNN, NB, and DT models, respectively. The ranking of the models' other performance metrics also shows parallelism with the classification success metric. As a result of the classifications performed with the active features selected by the BA, WOA, and GWO feature selection methods, the model with the highest classification success is mSVM. Again, NN, KNN, NB, and DT models are followed in the classifications carried out by the feature selection process. Likewise, the performance metrics of these models have similarities to their classification success. Consequently, it is seen that mSVM has the best classification performance from machine learning algorithms in the classification processes made as a result of deep feature extraction and feature selection.

As a result of the classifications performed with 1000 features obtained from the SqueezeNet model, it was seen that the highest classification success belonged to the mSVM model. As a result of the classifications made with the features obtained from the BA, WOA, and GWO feature selection methods, the highest classification success was obtained from the mSVM model, again. The ACC, TPR, TPR, PRE, F1-Score, MCC, and process time of these mSVM models are given in Table 4 and the graph showing the time taken for these classification processes is given in Figure 6.  Figure 7 gives the confusion matrix obtained as a result of the classification.

Figure 8 gives the performance metrics ACC, TPR, TPR, PRE, F1-Score, and MCC obtained as a result of the classifications performed with the mSVM, which has the highest classification success.

## 4. Conclusion

In this study, a feature vector containing 1000 deep features extracted from the images of four different corn types, BT6470, Calipos, Es_Armandi, and Hiva, by using the SqueezeNet model. Features were first classified by DT, NB, mSVM, KNN, and NN machine learning algorithms. Following, via BA, WOA, and GWO algorithms, more effective features selected from this feature vector were classified by DT, NB, mSVM, KNN, and NN machine learning algorithms. Finally, the performance results of the models were compared.

The performances of the classifiers were analyzed by using the confusion matrix data. The mSVM method achieved the highest classification performance in all classification processes performed with 1000 features obtained with the SqueezeNet, 480 features obtained with BA, 315 features obtained with WOA, and 384 features obtained with GWO. This model is followed by NN, KNN, NB, and DT methods in all classification processes, respectively. As a result of the classification of the feature vector obtained from deep feature extraction with mSVM, ACC, TPR, TPR, PRE, F1-Score, and MCC values were found to be 89.40%, 87.63%, 96.62%, 87.63%, 87.63%, and 84.24%, respectively. As a result of the classification of 480 feature vectors obtained by BA feature selection algorithm with mSVM, ACC, TPR, TPR, PRE, F1-Score, and MCC values were found to be 88.82%, 86.99%, 96.43%, 86.98%, 86.98%, and 83.41%, respectively. As a result of the classification of 315 feature vectors obtained by the WOA feature selection algorithm with mSVM, ACC, TPR, TPR, PRE, F1-Score, and MCC values were obtained as 88.72%, 86.89%, 96.40%, 86.86%, 86.87%, and 83.26%, respectively. Lastly, ACC, TPR, TPR, PRE, F1-Score, and MCC values were determined as 88.95%, 87.12%, 96.47%, 87.11%, 87.11%, and 83.58%, respectively, as a result of the classification of 384 feature vectors obtained by the GWO feature selection algorithm with mSVM.

## Figures and Tables

**Figure 1:** Sample corn seeds of four different types in the dataset.

**Figure 2:** A general convolutional neural network structure.

**Figure 3:** *k* = 10 cross validation used in the study.

**Figure 4:** Multi-class confusion matrix.

**Figure 5:** General block diagram of the study.

**Figure 6:** Comparison of mSVM models process time.

**Figure 7:** Confusion matrix of mSVM models.

**Figure 8:** Comparison of mSVM models performance metrics.

**Table 1:** Classification of some grain products with different artificial intelligence methods.

No	Crop	Accuracy (%)	Data pieces	Class	Method	References
1	Maize	99.13	1632	17	MLDA + LS-SVM	(Xia et al. 2019)
2	Maize	93.85	12,900	3	RBFNN	(Zhao et al. 2017)
3	Wheat maize	99.4	804	13	PCA + PLS_DA	(Sendin et al. 2019)
4	Maize	95.95	656	2	DCNN	(An et al. 2019)
5	Rice	93.02	3810	2	LR	(Cinar & koklu 2019)
6	Wheat	93.46	3000	2	ANN	(Kaya & saritas 2019)
7	Rice	88.07	200	3	CNN	(Ahmed et al. 2020)
8	Drybean	93.13	13,611	7	SVM	(Koklu & ozkan 2020)

**Table 2:** Parameters of the models used in the study.

Models	Parameters
mSVM	Cost (C): 1.00
	Regression loss epsilon (*Ɛ*): 0.10
	Regression cost (C): 1.00
	Complexity bound (v): 0.50 g: auto
	Numerical tolerance: 0.0010
	Iteration limit: 100
	Function: radial basis kernel

BA	Maximum frequency: 2
	Minimum frequency: 0
	Constant.alfa: 0.9
	Constant.gamma: 0.9
	Maximum loudness: 2
	Maximum pulse rate: 1
	Number of solutions: 10
	Maximum number of iterations: 100

WOA	Number of agents: 10
	Maximum number of iterations: 100
	Maximum frequency: 1
	Minimum frequency: 0
	Problem dimension: same as number of features

GWO	Alfa: 0,99
	Beta: 0,01
	Tres: 3
	Number of wolves: 10
	Maximum number of iterations: 100

**Table 3:** Comparison of classification performances for all model.

Feature selection method	Number of selected attributes	Classifier	Performance					
			ACC	TPR	TNR	PRE	F1-score	MCC
Deep feature extraction	1000	DT	70.59	66.73	90.54	66.77	66.74	57.24
		NB	72.15	68.35	91.05	68.71	68.40	59.52
		**mSVM**	**89.40**	**87.63**	**96.62**	**87.63**	**87.63**	**84.24**
		KNN	79.85	76.57	93.52	76.60	76.57	70.13
		NN	87.96	86.01	96.15	86.01	86.01	82.16

BA	480	DT	70.15	66.11	90.38	65.99	66.02	56.41
		NB	72.09	68.24	91.03	68.61	68.28	59.39
		**mSVM**	**88.82**	**86.99**	**96.43**	**86.98**	**86.98**	**83.41**
		KNN	79.87	76.58	93.53	76.65	76.57	70.16
		NN	87.38	85.32	95.96	85.32	85.32	81.28

WOA	315	DT	69.28	65.09	90.14	65.53	65.23	55.39
		NB	71.66	67.86	90.89	68.18	67.90	58.84
		**mSVM**	**88.72**	**86.89**	**96.40**	**86.86**	**86.87**	**83.26**
		KNN	79.61	76.31	93.45	76.33	76.31	69.79
		NN	87.26	85.16	95.92	85.20	85.18	81.10

GWO	384	DT	68.85	64.75	89.99	65.02	64.82	54.81
		NB	72.14	68.34	91.05	68.70	68.40	59.50
		**mSVM**	**88.95**	**87.12**	**96.47**	**87.11**	**87.11**	**83.58**
		KNN	80.12	76.84	93.61	76.91	76.85	70.51
		NN	87.30	85.20	95.93	85.23	85.21	81.15

**Table 4:** Performance metrics of mSVM models (%).

Method	Attributes	ACC	TPR	TNR	PRE	F1-score	MCC	Process time (sec)
Deep features + mSVM	1000	89.40	87.63	96.62	87.63	87.63	84.24	1604.4
BA + mSVM	480	88.82	86.99	96.43	86.98	86.98	83.41	614.3
WOA + mSVM	315	88.72	86.89	96.40	86.86	86.87	83.26	259.4
GWO + mSVM	384	88.95	87.12	96.47	87.11	87.11	83.58	418.7

## Data Availability

The data used to support the findings of this study are available from the corresponding author upon request.
